The article "Sentiment Analysis of Statements on Social Media and Electronic Media Using Machine and Deep Learning Classifiers" was retracted in 2023. Reasons: signs of a paper mill; suspected computer-generated content; unreliable results or conclusions; concerns about the data.

# Sentiment Analysis of Statements on Social Media and Electronic Media Using Machine and Deep Learning Classifiers

**DOI:** 10.1155/2022/9194031

**Published:** 2022-03-02

**Authors:** Anjali Goswami, Muddada Murali Krishna, Jayavani Vankara, Syam Machinathu Parambil Gangadharan, Chandra Shekhar Yadav, Manoj Kumar, Mohammad Monirujjaman Khan

**Affiliations:** ^1^Department of Mathematics and Statistics, College of Science and Theoretical Studies, Saudi Electronic University, Riyadh-13323, Saudi Arabia; ^2^Department of Computer Science & Engineering, Dr Lankapalli Bullayya College of Engineering, Visakhapatnam, Andhra Pradesh, India; ^3^Big Data Engineer, General Mills, Minneapolis, USA; ^4^Ministry of Electronics and Information Technology, Delhi, India; ^5^School of Computer Science, University of Petroleum and Energy Studies, Dehradun, Uttarakhand-248007, India; ^6^Electrical and Computer Engineering, North South University, Bashundhara, Dhaka-1229, Bangladesh

## Abstract

When it comes to our everyday life, emotions have a critical role to play. It goes without saying that it is critical in the context of mobile-computer interaction. In social and mobile communication, it is vital to understand the influence of emotions on the way people interact with one another and with the material they access. This study tried to investigate the relationship between the expressive state of mind and the efficacy of the human-mobile interaction while accessing a variety of different sorts of material over the course of learning. In addition, the difficulty of the feeling of many individuals is taken into account in this research. Human hardness is an important factor in determining a person's personality characteristics, and the material that they can access will alter depending on how they engage with a mobile device. It analyzes the link between the human-mobile interaction and the person's mental toughness to provide excellent suggestion material in the appropriate manner. In this study, an explicit feedback selection method is used to gather information on the emotional state of the mind of the participants. It has also been shown that the emotional state of a person's mind influences the human-mobile connection, with persons with varying levels of hardness accessing a variety of various sorts of material. It is hoped that this research will assist content producers in identifying engaging material that will encourage mobile users to promote good content by studying their personality features.

## 1. Introduction

Experiencing emotions is a necessary component of our everyday lives. They are there in everything we do, wherever we are, and everywhere we travel, and they do so without our even realizing they are there. Because we can see the other person's emotional expression on their face and because we do not receive an emotional reaction when we anticipate one, when it comes to mobile engagement, whether it is with people, technology, or humans through technology, all of us are suddenly more mindful of emotion. It is tough to distinguish between different emotions.

The article "Sentiment Analysis of Statements on Social Media and Electronic Media Using Machine and Deep Learning Classifiers" was retracted in 2023. Reasons: signs of a paper mill; suspected computer-generated content; unreliable results or conclusions; concerns about the data.

Emotions are complicated processes that are created by interactions between intentions, beliefs, perceptions, and circumstances, among other factors. To comprehend sentiments, we must, firstly, comprehend the mental state and situations of the person, as well as the sorts of processes that may be elicited by these conditions. The environment has an important part in determining the condition of the human mind. The human-computer/human-mobile interaction investigates the interaction between a person and a machine. It depends on supporting information from both the device and the human side [1]. A large number of scholars from throughout the globe have dedicated their careers to understanding the function of emotion in our interactions with technology.

In the field of affective computing [2–4], the research focuses on four main areas: (1) reducing user frustration, (2) enabling comfortable communication of user emotion, (3) developing infrastructure and applications to handle adequate information, and (4) developing tools that aid in the development of social and emotional skills.

This research seeks to determine the relationship between human emotional states and interaction, as well as to demonstrate that emotion has a greater impact on interaction than other factors. One of the primary goals of this research is to determine the relationship between human emotional states and interactions. As a result, it will aid the researcher in comprehending and inventing new techniques and technologies to realize the goal of affective computing as mentioned above. Our research team performed trials with real individuals who were interacting with different computer systems to evaluate this hypothesis, and they discovered the importance of the emotional state in human-computer interaction. In this experiment, the following are the goals that will be pursued.

The research begins by examining the many sorts of emotional states that people experience as a result of external events, challenges, and circumstances, as well as the impact these emotions have on their own life. Following up on the findings of the preceding research, we assume/fix other emotional scales for several additional events/problems/environments.

Secondly, we have divided events/situations into two categories: those that elicit good feelings and those that elicit negative emotions. The influence of good and negative emotions on human-computer interaction is also explored in more depth in this research.

The article "Sentiment Analysis of Statements on Social Media and Electronic Media Using Machine and Deep Learning Classifiers" was retracted in 2023. Reasons: signs of a paper mill; suspected computer-generated content; unreliable results or conclusions; concerns about the data.

The third part of our research looked at the influence of emotional mindset on human-computer interaction across a variety of interaction activities.

On a fourth level, we looked at how people react to certain emotional or mental states by looking into their own personal “hardness factor” and how that component affects them.

The fifth point is that the research examines the complete influence of stressful/festive events on human-computer interaction by comparing the average interaction impacts between the two groups of participants.

To conclude, to get fantastic content suggestions in understanding their mind-state and personality to modify their emotional level of a person is essential.

It is proposed to use the strategy of combining two (or more) procedures as a way of absorbing the benefits of both, and as a result, filling in some of the weaknesses of individual methods. Alfrjani and colleagues used a combination of machine learning and a semantic knowledge base to increase the accuracy of sentiment analysis on online reviews (an improvement from 1 percent to 6 percent). In another instance, a hybrid approach for sentiment analysis on tweets that incorporate both lexical and machine learning techniques (improvement: 2 percent to 6 percent). As a result, a hybrid system with collaborative features is better prepared to resolve any issues connected with a single system, if any such pitfalls exist. The efficiency of the integrated models may fluctuate depending on the job being performed. CNNs that have been upgraded by SVM, CNNs that have been enhanced by RNN, and Lexicon-based analysis with machine learning produced improved results. When doing sentiment analysis on diverse domains and kinds of datasets, the combination of CNN, LSTM, and SVM attempts to make use of the two deep network architectural models and SVM algorithms. There are also numerous sorts of input data that may be gathered via social networks, such as tweets and reviews, among other things. Within and across these forms of data, there are variations in the input data, such as the distribution of tweet and review durations, the variety of themes in each dataset, the sample size, and the higher or lower inclusion of explicit emotions and irrelevant information in each dataset. Some techniques may be unable to perform effectively over a range of domains, with poor accuracy and performance in sentiment analysis, for example. Specific procedures may be ill-suited and difficult to apply to certain kinds of input data as a consequence of this phenomenon.

The article "Sentiment Analysis of Statements on Social Media and Electronic Media Using Machine and Deep Learning Classifiers" was retracted in 2023. Reasons: signs of a paper mill; suspected computer-generated content; unreliable results or conclusions; concerns about the data.

One issue posed by our research is whether hybrid models outperform single models independent of the peculiarities of the datasets. Our findings suggest that they do. As a result, our research investigates the behavior of the chosen hybrid models when applied to various kinds of datasets from various domains. Using three different models, CNN, LSTM, and SVM, we investigated and verified their combination in this study. A link between the models and their increased capabilities to extract characteristics, retain previous information and nodes, and categorize text was studied. Firstly, in the early phases of the model, two potential variants in the sequence of CNN and LSTM are added, one for each of the two possible variations. Finally, two additional possibilities are presented for each of these options: the usage of CNN with ReLU function or SVM, and they are described in detail below. On eight datasets, including tweets and reviews, we tested these models with word embedding and found them to be effective. Using our research, we discovered that combining several models boosted the accuracy of sentiment analysis significantly.

Aside from highlighting four hybrid deep learning models for sentiment analysis that produce improved accuracy regardless of the types of social network datasets used, this paper also provides an experimental study to evaluate the performance of hybrid deep learning models and details a performance comparison of sentiment analysis methods with some state-of-the-art methods, all of which are significant contributions to the literature.

In the wake of our investigation, we have discovered that emotional mentality plays an important role in human-computer/mobile-interface interaction. Apart from that, the toughness factor of individual users might be either good or bad, depending on their experience. This element has an influence on the interaction between humans and computers or mobile devices. Whenever the hardness factor is positive, the emotional mentality has only a little influence on human-computer/mobile interaction activities. At the same time, when the emotional aspect has a stronger impact on the interaction task, the hardness factor has a negative effect. Consequently, according to their hardness level, the user receives varied material suggestions to replicate happy feelings in their minds, which will cause them to be more optimistic and help them to operate more productively in their settings.

The remainder of the paper is organized according to the arrangement outlined subsequently.  Section 2 examines the most important techniques in human-emotion-based literature, as well as the most typical works in this area of study. In the third page, we talk about the significance of human emotion and the many emotional mindsets that a typical human being has under different situations. It categorizes both good and negative emotions, as well as events or circumstances that elicit either positive or negative emotions in the participant.  Section 4 goes to great lengths on the emotional difficulties that are investigated experimentally.  Section 5 delves into the relationship between mobile interaction suggestions and other variables in more depth than the previous sections. A summary of the lessons we have gained is provided in Section 6. The aspects of system development that are influenced by emotion are discussed in Section 7, as is the inclusion of emotional information into system development. Section 8 describes the process of suggestion for transforming negative emotional states into good emotional states. Finally, Section 9 summarizes our findings and our plans for the future.

The article "Sentiment Analysis of Statements on Social Media and Electronic Media Using Machine and Deep Learning Classifiers" was retracted in 2023. Reasons: signs of a paper mill; suspected computer-generated content; unreliable results or conclusions; concerns about the data.

## 2. Literature Survey

Consider the significance of employing current technology tools in everyday life and how much effort has been done to provide answers to practical computing throughout the globe. Because of the arrival of Android technology, microcomputer system developers gained a fresh perspective, and a slew of new apps were built. This section examines the many research projects that have been undertaken in this field, as well as the creation of successful computing-based solutions.

Michigan Technological University's Myounghoon Jeon published a chapter in the book “Foundations of Affective Sciences” in 2017, titled “Emotions and Affect in Human Factors and Human-Computer Interaction: Taxonomy, Theories, Approaches, and Methods,” in which he surveyed several approaches of Affective Science in Human Factors/Human-Computer Interaction. Their backgrounds, objectives, and approaches are all distinct. However, all of them clearly demonstrate that emotions and affect are not ancillary, but rather one of the fundamental aspects in Human Factors/Human-Computer Interaction design, and they all attempt to integrate all of the techniques to achieve effective results. By bridging the gap between conventional Human Factors/Human-Computer Interaction research and the new subject of Affective Sciences research, this handbook helps each discipline advance its own knowledge and understanding.

Researchers from Michigan Technological University published a chapter in the book “Fundaments of Affective Sciences” in 2017 called “Neural Mechanisms of Emotions and Affect,” in which they reviewed many capabilities and components of the brain's functioning in depth. 3. Jacob Aday comes to the conclusion that emotion is not a single process and that the emotional brain is not a specific area of the brain. Emotions are multistage, complicated events, and the brain representation of them is distributed and connected to the stage of emotional processing at which they occur.

The article "Sentiment Analysis of Statements on Social Media and Electronic Media Using Machine and Deep Learning Classifiers" was retracted in 2023. Reasons: signs of a paper mill; suspected computer-generated content; unreliable results or conclusions; concerns about the data.

According to Hillary A. Elfenbein et al., this paper explores the social perception of emotional intelligence and extends the data to assess its reliability and cross-judge agreement, as well as its convergent, divergent, and predictive validity, among other factors. Although several parameters were taken into consideration, the observation research nevertheless showed a substantial correlation with interdependent task performance. Notably, the predictive validity of observer-rated emotional intelligence was higher than that of self-rated or ability-tested emotional intelligence.

The fourth point to mention is that, in the year 2019, Sam Freed's chapter “Prevailing Prejudices About Artificial Intelligence” in the book “AI and Human Thought and Emotion” shows that some outdated ideas, opinions, attitudes, and metaphors have had an impact on cognitive science and Artificial Intelligence (AI), despite the fact that there is insufficient evidence to support their claims. It delineates some of the underlying assumptions that support much of our culture, and in particular, much of artificial intelligence research and development.

“Artificial intelligence for affective computing: an emotion recognition case study,” by Pablo Arnau-González and colleagues, provides an introduction to the benefits of artificial intelligence techniques for the field of affective computing through a case study about emotion recognition via brain (electroencephalography-EEG) signals. Pablo Arnau-González and colleagues' chapter “Artificial intelligence for affective computing: an emotion recognition case study” is available online. It was discovered that artificial intelligence-based systems for emotion identification have great potential, as shown by the data collected. There is great potential for this application to make a significant contribution to the fields of human-computer interaction (HCI) and quality of experience (QoE).

In 2008, Brian R. Duffy, a professor at the Massachusetts Institute of Technology, stressed the need of automating emotion to regulate systems at various levels.

In a 2004 paper, Antonella De Angeli and Graham I. Johnson pointed out that computational reductionism has led to an inaccurate perspective of emotions, which thinks that they are only physical and cognitive, however, they are really deeply anchored in social contexts.

The article "Sentiment Analysis of Statements on Social Media and Electronic Media Using Machine and Deep Learning Classifiers" was retracted in 2023. Reasons: signs of a paper mill; suspected computer-generated content; unreliable results or conclusions; concerns about the data.

In 2005, Jackeline Spinola de Freitas emphasized the need for emotion design to accurately express emotions. Nevertheless, no comparison was made between emotional and nonemotional systems. Furthermore, it is vital to establish techniques for recording emotional experiences to better understand them.

The multicomponent approach to emotions proposed by Scherer [5] was highlighted in a 2006 study from the Berlin University of Technology, in which different aspects of emotions in an interactive context were investigated: subjective feelings, physiological activation, motor expression, cognitive appraisals, and behavioral tendencies [6–8]. It was discovered that the quality of use differed between two versions of an interactive system that used different emotional states in different ways. Researchers discovered that systems with high usability provide more positive sentiments than systems with usability problems, according to the results of the research. There are a range of ways that may be used to discover differential variations, including rating scales for subjective feelings, electromyography (EMG) of muscle activity in the face, heart rate, ECG (EDA), performance data, and questionnaires for cognitive evaluations. Additionally, it was hypothesized that this combination would provide an extensive framework to comprehend emotional expressions in human-computer interaction (HCI).

In 2018, Jackeline Spinola de Freitas and colleagues aimed to examine the recording of emotions using a number of approaches, including audios, videos, and explicit procedures, to better understand the phenomenon. Each design makes no effort to evaluate or analyze the human harness or the mental state of the subject. Therefore, new approaches for capturing emotional states, as well as fundamental sentiments, are necessary, according to the findings of the study. Our mission is to create a new Android application that will assist scientists in gaining access to emotional mind states, human hardiness, and situation-specific emotions, among other things.

Kövecses analyzes the eleventh in the year 2018. According to the author, conceptual metaphors may be employed to frame media discourses both intratextually and intertextually, and they can be utilized both ways. However, they may also be able to explain what seems to be incoherent media speech, which appears to be the norm in the majority of instances. The idea of conceptual metaphor contributes to our understanding of why people instinctively blend metaphors. As a result of the priming effect, the context in which media discourse is presented has a significant impact on how effective it is. A variety of practical considerations make headlines, especially vulnerable to the contextual impact in their content in particular. Finding noteworthy patterns in media discourse may be accomplished by recording the structure of this cognitive process and then analyzing it. In this essay, the author argues that metaphors should be used to express the meaning of the activities that are being done.

The article "Sentiment Analysis of Statements on Social Media and Electronic Media Using Machine and Deep Learning Classifiers" was retracted in 2023. Reasons: signs of a paper mill; suspected computer-generated content; unreliable results or conclusions; concerns about the data.

According to Kövecses, in his book titled, “Where Metaphors Come from: Reconsidering Context in Metaphor,” he describes the desire for happiness as a metaphor and how to apply it in different information processing settings in the chapter headed, “Happiness in Context”.

When it comes to understanding human well-being, the authors of “Emotion in the Digital Age: Technologies, Data, and Psychosocial Life” (Emotion in the Digital Age: Technologies, Data, and Psychosocial Life, published in 2021) stress the need for dynamic modeling and knowledge. Also emphasized is the idea that this constitutes a psycho-social style of being, in which digital technology and emotion function as significant parts of the method in which we simultaneously connect to ourselves as individual subjects and to others as the members of collectives.

The relevance of synthetic cognitive emotions in the design of robot-based systems is highlighted by Jordi Vallverdi (2016) in his article. According to him, it is one of the most significant elements in the design of complex systems.

According to F. Gregory Ashby of the University of California, Santa Barbara's positive effect hypothesis, which was created in 1999, pleasant emotion enhances performance on a broad variety of cognitive tasks. Several contemporary neuropsychological hypotheses propose that pleasurable feeling is associated with increased dopamine levels in the brain, which, according to the theory, would account for many of these benefits. It predicts or accounts for the impacts of positive emotion on olfaction, long-term (i.e., episodic) memories, working memory, and the capacity to solve creative issues, to name a few aspects.

Dr. Barbara L. Fredrickson's research in 2018 is focused on positive emotions and psychophysiological laboratory to develop a data-driven model from the bottom up. It describes how individual heterogeneity in immune, parasympathetic, and oxytocin profiles manifests itself in different situations. Furthermore, it serves as a foundation for individual variations and good feelings. She utilizes the word “purpose” as an umbrella phrase to embrace these diverse types of self-transcendence because it is both accessible and alliterative with good feelings and because it is both accessible and alliterative with positive emotions. A major emphasis of the author's research is on possible biological processes via which pleasant mental states, such as happy emotions and a sense of purpose, might be connected to physical health over time. The broaden-and-build hypothesis serves as a theoretical framework for investigating the biological bases of positive feelings and intentions, as well as their consequences. Then, pleasant emotions and a sense of purpose are dynamically connected, and each seems to play a crucial role in regulating the leukocyte gene expression, which appears to be a reasonable biological substrate of living a fulfilling life.

The article "Sentiment Analysis of Statements on Social Media and Electronic Media Using Machine and Deep Learning Classifiers" was retracted in 2023. Reasons: signs of a paper mill; suspected computer-generated content; unreliable results or conclusions; concerns about the data.

Denis Rangulov and Muhammad Fahim created a method to detect the emotions shown in video clips in the year 2020. When predicting dimensional emotions from video data, the system model design model blends a convolutional neural network (CNN) with a recurrent neural network (RNN). CNN begins by extracting feature vectors from video frames in the first stage. In the second phase, we input these feature vectors into an RNN that was being trained to exploit the temporal dynamics of video. In addition, we looked at how each neural network contributed to the overall performance of the system in question.

It is crucial, according to Tianyi Zhang et al., 2021, to try to discern user emotions when viewing short-form videos at any time and from any location. It will allow for video content customization and personalization. However, the majority of the studies either categorize a single emotion per video stimulus or confine it to static, desktop surroundings. It made use of wearable gadgets to track the emotions of participants.

In a study published in 2020, Shihan Ran and colleagues sought to detect emotions using electroencephalography (EEG)-based emotion identification. Their work has improved the area of affective computing and allowed applications in human-computer interactions. The decoding of emotion using supervised machine-learning algorithms has advanced significantly in recent years, while other research have used data-driven, unsupervised methodologies to investigate the underlying EEG patterns during an emotion experiment. It investigates the relationship between such dynamics and subjective assessments of emotion.

Researchers S. Hsu et al. observed in 2018 that a better knowledge of how neurocognitive processes affect hypnotherapy may enhance therapeutic results. When continuous electroencephalographic (EEG) data captured under hypnosis is used to decode cortical state changes, it presents a significant difficulty. We use adaptive mixture independent component analysis (AMICA) to predict changes in the brain state dynamics during hypnosis. AMICA is an unsupervised technique that trains many independent component analysis models for defining nonstationary, unlabeled data. The application of the AMICA model to EEG data from six hypnosis sessions revealed changes in system-wide brain activity that corresponded to transitions between hypnosis levels. The findings also revealed that AMICA-based models were constant across sessions and participants and that they mirrored diverse patterns of source activity in various hypnosis stages as a consequence. Changes in the theta, alpha, and other spectral properties of source activity were identified during the treatment sessions via the analysis of independent component clusters associated with separate classes of model probability patterns.

The article "Sentiment Analysis of Statements on Social Media and Electronic Media Using Machine and Deep Learning Classifiers" was retracted in 2023. Reasons: signs of a paper mill; suspected computer-generated content; unreliable results or conclusions; concerns about the data.

Banzige (2009) from the Geneva University indicated that emotion detection capacity is a critical component of emotional competence and is a core component of emotional intelligence. Aim: to develop a tool that objectively assesses this ability using actor portrayals of dynamic expressions of 10 emotions (2 variants each for five emotion families), operationalized as recognition accuracy in four presentation modes that combine the visual and auditory sense modalities (audio/video, audio-only, video-only, and still picture). The many experiments and the usefulness of a test design are used to assess coarse and fine-grained emotion discrimination and modality-specific abilities in children. The results of the factor analysis indicate that there are two distinct talents, namely visual recognition and aural recognition, that seem to be substantially independent of personality dispositions.

The preceding works demonstrate that all of these studies instantaneously capture the emotions using a variety of approaches, including audios, movies, and explicit methods, among others. None of these studies took into account the consumers' attitude or level of difficulty. As a result, this work takes into account the consumers' point of view as well as their genuine circumstances and basic feelings. It will provide more effective outcomes, as seen by this work in progress. It also aids in the recommendation of more interesting information to consumers.

As a field, affective computing exists at the intersection of artificial intelligence and human-computer interaction design. “To understand human emotions and give robots feelings, “emotional modules” will be added to rule-based artificial intelligence systems,” the researchers said. The field is seeing unprecedented growth in popularity. A new generation of wearable computers equipped with physiological sensors and pattern recognition is being developed to collect and analyze signals that are intended to communicate the user's emotional state [1, 9].

The article "Sentiment Analysis of Statements on Social Media and Electronic Media Using Machine and Deep Learning Classifiers" was retracted in 2023. Reasons: signs of a paper mill; suspected computer-generated content; unreliable results or conclusions; concerns about the data.

Scientists are concentrating their efforts on emotion-based computational architectures [8], whose models physiologically inspire the emotion process explored by neuroscience, allowing them to include emotions into machines' functions control or generate an “artificial emotion.” According to widespread expectations, adding an emotion model in the computational system would increase machine performance in areas, such as decision-making competence, action selection and control, and autonomous and reliable system response. Human emotion understanding, learning, and measurement collect information about a user's emotional state during an encounter with the user, allowing for the provision of appropriate help or services that are tailored to the user's requirements. A user's emotional requirements are recognized, and providing those needs is likely to result in a satisfactory connection with that user. It is the motivation for human emotion learning. Although it is difficult to comprehend and model human emotions, it is possible to organize and quantify the intensity of emotion experienced by a person when engaging with a system [10–14].

It is necessary to identify significant patterns from the collected data to recognize emotional information [15–18]. Various algorithms, such as voice recognition, natural language processing, and facial expression detection, are used to parse the data, all of which are based on the human component rather than programming, and hence, they need human intervention [19]. We study emotional learning in the context of a mixed-initiative interaction [19], in which the system alters its behavior or function in response to the user's mood. The most typical technique to developing an emotional system is to learn about the user's emotional state and then operate the system in a variety of different modes. We aimed to investigate the link between human emotion and computer interaction in this research.  Table 1 represents the parameter of the input data set.

In accordance with their emotional state, each individual works and interacts with the system in a distinct manner [20–22]. Consequently, it is reasonable to assume that each user will engage with the system in a personalized manner. As a result, the kind of support a user desires and the activities a user expects from the system alter, depending on the user's emotional state. In the case of a particular user who is under a lot of stress, he or she may choose to relax for a few hours or do anything monotonous. As a result of the system's improved emotional awareness of the user, the system provides new means of engagement in response [23]. When the user is under extreme stress, the system may instruct him or her to work in safe mode. In the same manner, we must recognize and respond to the emotional states of various users to adjust the system's engagement with them appropriately [24].

The article "Sentiment Analysis of Statements on Social Media and Electronic Media Using Machine and Deep Learning Classifiers" was retracted in 2023. Reasons: signs of a paper mill; suspected computer-generated content; unreliable results or conclusions; concerns about the data.

Briefly, the significance of emotional learning rests in its ability to enable the user to provide free input while engaging with the system. The next section explains the range of human emotional states and their implications when dealing with a system [25], which should be taken into account while designing new tactics for engaging with it. It is also necessary to find new technologies and procedures for determining the emotional condition of people [26].

## 3. Model System Design for Sentiment Analysis while Video Playing

There are two possible outcomes for the data:

  It may be regarded as expressing which movies the users have seen (and rated) and which films they have not watched. In this case, users' timepieces serve as a type of tacit feedback, letting us know which items they want to view and which they would rather not see.
  It may also be seen as a way of expressing how much the users enjoyed the films that they did view. It is an example of explicit feedback: assuming that a person has viewed a movie, we can infer how much they enjoyed it by looking at the rating they have given to the film.

An android mobile app is designed and developed to play the videos in it. In this system, the mobile app is designed to recommend different videos to the users. Based on their experience, the user instructs the other video contents to other users. The system design asks a different question when watching the video [27], and the user is giving the answers. By considering this feedback, the users are classified into different categories. The factors taken for the classification of users are as follows: 1) mindset, 2) human hardness, 3) positive emotion, and 4) negative emotion. Now, it will make a recommendation using the following KNN algorithm. The complete details of the KNN algorithm are presented in the latter part of this section. In this work, we have done a further analysis of different personalities and their recommendations for consideration. The effectiveness of these recommendations is analyzed to understand the relativity between the personality types and their recommendations [28].  Figure 1 depicts how the human mobile video content accessing architecture shows how video content accesses from live video streaming.  Figure 2 shows a snapshot of a video mobile video app.

We divided the dataset into two groups: training sets and test sets. The following function offers two split modes, one of which is random and the other one is seq-aware. If one chooses the random mode, the function divides the 100k interactions randomly without taking into account the timestamp, and by default, it utilises 90 percent of the data as training samples and the remaining 10 percent of the data as test samples. In the seq-aware mode, we exclude the item that a user has rated the most recently from the test, as well as the users' previous interactions from the training set. The historical interactions of users are arranged from the oldest to the newest, depending on the timestamp of their interactions. It will be utilized in the sequence-aware recommendation phase of the Algorithm 1.

The article "Sentiment Analysis of Statements on Social Media and Electronic Media Using Machine and Deep Learning Classifiers" was retracted in 2023. Reasons: signs of a paper mill; suspected computer-generated content; unreliable results or conclusions; concerns about the data.

Eight textual tweets and review datasets from diverse fields are used to train and evaluate hybrid deep sentiment analysis learning models that integrate long short-term memory (LSTM) networks, convolutional neural networks (CNN), and support vector machines (SVM).

Each user profile is a combined group of emotional attributes that will be modeled as Ux = {Ex1, Ex2, Ex3, Ex4, Ex5}, where “Ex” represents the emotion status of the user, i.e., Ex1 is representing the hardness factor, Ex2 is representing the stress factor, Ex3 is representing the positive emotion factor, Ex4 is representing the negative emotion factor, and Ex5 is representing positive thinking/negative thinking factor [29]. The contents are selected based on the user's relation with the user and the movies.

In this experimentation, the IMDb Dataset is taken for experimentation. It is a dataset available for access to customers for personal and noncommercial use. The IMDb Movie Reviews dataset is a binary sentiment analysis dataset consisting of 50,000 reviews from the Internet Movie Database (IMDb) labeled as positive or negative. The dataset contains an even number of positive and negative reviews. Only highly polarizing reviews are considered. It is further tuned to meet our requirements in this work.

The performance of the proposed recommendation scheme is evaluated based on the evaluation metrics of accuracy, precision, recall, and F-measure [30]. The accuracy metrics are defined as the potential in predicting labels associated with a categorical class. In other words, it is computed as the proportion of correctly predicted instances as specified in (1).

(1) $$\begin{array}{c} \mathrm{Accuracy=}\frac{\mathrm{True}\;\mathrm{Positive+True}\;\mathrm{Negative}}{\mathrm{True}\;\mathrm{Positive+True}\;\mathrm{Negative+False}\;\mathrm{Positive+False}\;\mathrm{Negative}}. \end{array}$$

Precision refers to the closeness measures of instances with one another, and it is computed based on (2).

(2) $$\begin{array}{c} \mathrm{Precision=}\frac{\mathrm{True}\;\mathrm{Positive}}{\mathrm{True}\;\mathrm{Positive+False}\;\mathrm{Positive}}. \end{array}$$

Recall is defined as the exact positive instance in the dataset that has been accurately determined as positive by the utilized classifier [31], as calculated based on (3).

(3) $$\begin{array}{c} \mathrm{Recall=}\frac{\mathrm{True}\;\mathrm{Positive}}{\mathrm{True}\;\mathrm{Positive+False}\;\mathrm{Negative}}. \end{array}$$

In addition, the *F*-Measure is computed based on the weighted harmonic mean of the recall and precision as mentioned in (4).

(4) $$\begin{array}{c} \mathrm{F-}\mathrm{Measure=}\frac{\mathrm{2\times Precision\times Recall}}{\mathrm{Precision+Recall}}, \end{array}$$

TP (true positive): if the instance is positive and the outcome of the predicted recommendation is also positive. TN (true negative): if the instance is negative and the outcome of the predicted recommendation is also negative [32]. FN (false negative): if the record is positive and the outcome of the predicted recommendation is also negative. FP (false positive): if the data record is negative and the outcome of the predicted recommendation is also positive.

The article "Sentiment Analysis of Statements on Social Media and Electronic Media Using Machine and Deep Learning Classifiers" was retracted in 2023. Reasons: signs of a paper mill; suspected computer-generated content; unreliable results or conclusions; concerns about the data.

## 4. User-Interaction Emotional Issues: Empirical Study

The goal of our experiment was to study different aspects of the recommendations between a user and the mobile under various mindsets. Specifically, we learned classified different types of events/situations that evoked positive and negative emotions. Furthermore, the study extends the impact of positive and negative feelings in human-mobile interaction. Besides, we studied various critical aspects of human hardness to estimate the average interacting capacity [33]. This section is organized as follows: Section 4.1 describes our experiment participants' characteristics and background.  Section 4.2 describes our experiment procedure. Finally, Section 4.3 presents the results we have obtained.

### 4.1. Experiment Participants

Thirty users ranging in age from 19 to 45 years—14 male and 16 female—participated in the experiment. Five different categories of participants, such as 1. Sports Videos Watchers (23%), 2. Movie Videos Watchers (13%), 3. Social Video Watchers (20%), 4. Student/Learner Videos Watchers (17%), and 5. Medical/Professional/Business Man Content Watchers (27%). These video watchers have specifically watched a set of videos in Table 2, and Figure 1 shows the percentage.

We categorized the first group of participants as hard personality (37%), the second group as moderately hard personality (43%), and the last group of participants as low-hard personality (20%).  Figure 2 shows the personality traits survey done using one-time questionnaire by a professor from the University of Chicago.

The article "Sentiment Analysis of Statements on Social Media and Electronic Media Using Machine and Deep Learning Classifiers" was retracted in 2023. Reasons: signs of a paper mill; suspected computer-generated content; unreliable results or conclusions; concerns about the data.

### 4.2. Experiment Procedure

All participants were given a survey with questions regarding their mindset at the beginning of playing the videos and the performance after watching the videos. The users were asked to answer the questionnaire providing as much information as possible. We consider all kinds of answers to be equally important and valuable for our study since we want to know how the different users feel about watching videos. The user is permitted to recommend a set of videos to the other users. The effectiveness of the user recommendation is measured and studied in this work.

### 4.3. Experiment Results

The following sections describe in detail the results we have obtained from our experiment. How does human hardness impact human-mobile interaction? Each section addresses a particular issue regarding human hardness and emotional states in user interaction. Based on their hardness level, different videos were recommended in understanding the personality.

#### 4.3.1. Does Human-Hardness Impact the Human-Computer Interaction?

Each person has a different personality and interacts with the system in a certain way. The hardness of each person differs because of other reasons. Other methods are available for measuring the user's mental status [11, 12, 14, 34]—the technique of hardness assessment is given in Annexure-A. For example, some people are with high hardness, while some people have low hardness. The average interaction score is fixed for each type of interaction task, and such a score converts to an average score of 10. Then, based on the hardness score, the users classify into three categories, namely the high-hardness person, moderate hardness person, and low-hardness person. Their recommendation considers attributes, such as accuracy, precision, recall, and F1-measures, plotted in the following Figures 3–7. It is observed that the high-hardness persons have a good level of recommendations compared with those of moderate hardness and low hardness. It established that the hardness aspect of the system plays a vital role in the mobile/computer-human interaction. Therefore, human hardness increases, and there is a high interaction performance.  Table 3 includes the average mobile interaction score.

#### 4.3.2. Does Stress Impact Human-Computer Interaction?

Each person has different encounter situations in everyday life, and the conditions and events change the stress rate of the person. Annexure B gives the list of stress events and their rating, and each person has a different stress rate than their computer/mobile-interaction efficiency on two additional days. The stress rate readjusts to the given hardness and interaction values. Then, based on the stress score, the user classification is carried out into two categories. One is the person with high stress and the person with low-stress, and their recommendation considers attributes, such as accuracy, precision, recall, and *F*1-measures plots, in the following Figures 8–11. It observes that the low-stress persons are having a good level of recommendations compared with high-stress persons.

The article "Sentiment Analysis of Statements on Social Media and Electronic Media Using Machine and Deep Learning Classifiers" was retracted in 2023. Reasons: signs of a paper mill; suspected computer-generated content; unreliable results or conclusions; concerns about the data.

#### 4.3.3. Does Positive Emotion Impact Human-Computer Interaction?

Each person is encountering different situations in day-to-day life. The conditions and events change the emotional status of the person. Each person with different positive emotional levels is asked to present their emotional status twice or thrice a day for a particular period. Its average compares with their recommendations efficiency. Based on the positive emotion score, the users are classified into two categories. One is the person with high-positive emotion and the other is the person with low positive emotion. Their recommendation considers that the high-positive feelings persons have a good level of requests compared with high-stress persons. Appendix C presents the list of positive emotional events, and their ratings as shown in Figures 12–15).

#### 4.3.4. Does Negative Emotion Impact Human-Computer Interaction?

Each person has seen a different situation in everyday life. The situations and events change the emotional status of the person. Appendix-D presents the list of negative emotional events and their rating. Each person with different harmful emotional levels was asked to explain their emotional situation twice or thrice a day for a particular period. Its average compares with their recommendations efficiency. Based on the negative emotion score, the users are classified into two categories. One is the person with high-negative emotion. The person with low negative emotion and their recommendations consider attributes, such as accuracy, precision, recall, and *F*1-measures plots, in the following Figures 16–19. It observes that the low-negative emotion persons have a good level of recommendations compared with those of high-negative emotional people.

#### 4.3.5. Does Positive Thinking Impact Human-Computer Interaction?

Each person has a different personality and interacts with the system in a certain way. The positive attitude of each person differs because of various reasons. Annexure-E presents the method of attitude assessment. For example, some people have a high positive thinking attitude, and some people have a low positive thinking attitude. The score is fixed for the average interaction for each interaction task, and such a score converts to an average score of 10. Then, the average actual observed interaction performance is compared to the positive thinking attitude score and is presented in the following Figure 7.

The article "Sentiment Analysis of Statements on Social Media and Electronic Media Using Machine and Deep Learning Classifiers" was retracted in 2023. Reasons: signs of a paper mill; suspected computer-generated content; unreliable results or conclusions; concerns about the data.

The following table presents the simple correlation between the interaction and between the attributes compared.  Table 4 represents the correlation details.

Let AC, HD, ST, PE, NE, and PT be represented by *X*1, *X*2, *X*3, *X*4, *X*5, and *X*6, respectively, since *X*1 is dependent on *X*2, *X*3, *X*4, *X*5, and *X*6. We take the measurements of these variables from their expected values. Consequently,

(5) $$\begin{array}{c} E\left(X1\right)=0=E\left(X2\right)=E\left(X3\right)=E\left(X4\right)=E\left(X5\right)=E\left(X6\right). \end{array}$$

Let the standard deviation be *σ*_1_, *σ*_2_, *σ*_3_, *σ*_4_, *σ*_5_, and *σ*_6_. Let the correlation between these variables be **r**12, **r**13, **r**14, **r**15, **r**16, **r**23, r24, **r**25, **r**26, **r**34, **r**35, **r**36, **r**45, **r**46, and **r**56.

It is possible to determine the plane of regress of *X*1 in terms of *X*2, *X*3, *X*4, *X*5, and *X*6, and it is given by the following:

(6) $$\begin{array}{c} \left(\frac{X1}{\sigma_{1}}\right)\omega 11+\left(\frac{X2}{\sigma_{2}}\right)\omega 12+\left(\frac{X3}{\sigma_{3}}\right)\omega 13+\left(\frac{X4}{\sigma_{4}}\right)\omega 14+\left(\frac{X5}{\sigma_{5}}\right)\omega 15+\left(\frac{X6}{\sigma_{6}}\right)\omega 16=0,\\ \omega =\left[\begin{array}{cccccc} 1 & r_{12} & r_{13} & r_{14} & r_{15} & r_{16}\\ r_{21} & 1 & r_{23} & r_{24} & r_{25} & r_{26}\\ r_{31} & r_{32} & 1 & r_{34} & r_{35} & r_{36}\\ r_{41} & r_{42} & r_{43} & 1 & r_{45} & r_{46}\\ r_{51} & r_{52} & r_{53} & r_{54} & 1 & r_{56}\\ r_{61} & r_{62} & r_{63} & r_{64} & r_{65} & 1 \end{array}\right]\left[\begin{array}{cccccc} 1 & r_{12} & r_{13} & r_{14} & r_{15} & r_{16}\\ r_{21} & 1 & r_{23} & r_{24} & r_{25} & r_{26}\\ r_{31} & r_{32} & 1 & r_{34} & r_{35} & r_{36}\\ r_{41} & r_{42} & r_{43} & 1 & r_{45} & r_{46}\\ r_{51} & r_{52} & r_{53} & r_{54} & 1 & r_{56}\\ r_{61} & r_{62} & r_{63} & r_{64} & r_{65} & 1 \end{array}\right]. \end{array}$$

We note here that the corresponding cofactor of the element in the *i*^th^ row and *j*^th^ column is *ωij* for all *i*, *j* ranging from 1 to 5.

The coefficient of multiple correlations in six variate distributions in which each of the variables *X*1, *X*2, *X*3, *X*4, *X*5, and *X*6 in terms of the mutual correlations between *i*, *j* is given by the following:

(7) $$\begin{array}{c} R_{1.23456}^{2}=1-\frac{\omega }{\omega_{11}}. \end{array}$$

The coefficient of multiple correlations estimates the closeness of association between the observed values and the expected value of a variable obtained from the multiple linear regression of that variable on other variables.

The article "Sentiment Analysis of Statements on Social Media and Electronic Media Using Machine and Deep Learning Classifiers" was retracted in 2023. Reasons: signs of a paper mill; suspected computer-generated content; unreliable results or conclusions; concerns about the data.

*R*_1.23456_^2^ is a simple correlation between *X*1, and the error estimate *e*_1_ is 0.23456. It must lie between −1 and +1. However, in our case, it will be 0 ≤ *R*_1.23456_^2^ ≤ 1. It establishes that the correlation between the hardness and accuracy is highly correlative. Therefore, it is considered to be one of the important attributes taken for analysis.

## 5. Experimental Learning

The experiment showed several fascinating features of an emotion's influence in human-computer interaction. Computer systems or software systems have been unable to personalize or comprehend the user's emotions. We observed several challenges that exchange-system designers must address to personalize and optimize the interaction system and users.

- Understand the relation between user interaction and the hardness of the person.
- Understand the relation between user interaction and the stress rate of the person.
- Understand the relation between user interaction and the positive emotion of the person on a particular day.
- Understand the relation between user interaction and the negative emotion of the person on a particular day.
- Understand the relation between user interaction and the positive thinking attitude of the person.
- Discovering the method for providing implicit feedback to capture these attributes.
- Discovering the new method of mobile interaction mechanisms to each set of users.

## 6. Implications in Human-Emotional System Development: How to Incorporate Emotional Knowledge

To provide better interaction to the computer user, the system needs some emotional knowledge about them. Now, this knowledge is collected through explicit feedback. However, we need to develop new devices, mechanisms, and methods to manage these knowledge sets automatically. The most crucial fact about human emotion is that it is both instantaneous and intrinsic. Our approach analyzes the people's relativity hardness, stress, positive emotion, negative emotion, and positive thinking attitude. It is hard to understand the positive and negative emotions because it is instantaneous. The system uses four ways to collect emotional details. The first method is to observe the user's emotional status through the new hardware devices, utilizing relative measures like blood pressure. The second method is to identify facial expressions, and the third method is to collect explicit feedback from the user. The fourth method is information personalization. A commonly used metaphor for accepting the user's emotional status is consuming a personal assistant interface-agent collaborating with the user in some work environment. Over some time, the system will acquire a complete emotional attitude of the user.

The article "Sentiment Analysis of Statements on Social Media and Electronic Media Using Machine and Deep Learning Classifiers" was retracted in 2023. Reasons: signs of a paper mill; suspected computer-generated content; unreliable results or conclusions; concerns about the data.

In general, users' emotional information can be fed to the system, and it is possible to adapt the user for both system and application software development cases. All these emotional statuses are kept under the category of the application-independent information domain.

## 7. Conclusions

This paper has studied the relativity between user interaction and emotional attributes, such as hardness, stress, positive emotion, negative emotion, and positive thinking. The study presented the results of an experiment to learn the impact of incorporating emotional knowledge into the system.

This work gives an idea about the understanding of user-emotion status while interacting with the system. This study has implications on designing an interface with emotional knowledge to improve the system's overall efficiency. There are seven significant issues for the incorporation of emotional understanding, which are as follows:

- Understand the relation between user interaction and the hardness of the person.
- Understand the relation between user interaction and the stress rate of the person.
- Understand the relation between user interaction and the positive emotion of the person on a particular day.
- Understand the relation between user interaction and the negative emotion of the person on a particular day.
- Understand the relation between user interaction and the positive thinking attitude of the person.
- Discovering the method for providing implicit feedback to capture these attributes.
- Discovering the new method of machine interaction mechanisms to each set of users.

We have developed techniques for learning and incorporating emotional information to address the issues outlined above. We are also focusing on dynamic user profile techniques that analyze user interactions to determine emotional user status. One can use the results of these algorithms in future systems.

## Figures and Tables

**Figure 1:** Human mobile interaction system in accessing video contents.

**Figure 2:** A snapshot of Video Mobile App.

**Figure 3:** Accuracy measure of different human hardness of recommendations.

**Figure 4:** Precision measure of different human hardness of recommendations.

**Figure 5:** Recall measure of different human hardness of recommendations.

**Figure 6:** Accuracy measure of different stress level of recommendations.

**Figure 7:** Precision measure of different stress level of recommendations.

The article "Sentiment Analysis of Statements on Social Media and Electronic Media Using Machine and Deep Learning Classifiers" was retracted in 2023. Reasons: signs of a paper mill; suspected computer-generated content; unreliable results or conclusions; concerns about the data.

**Figure 8:** Recall measure of different stress level of recommendations.

**Figure 9:** *F*1 measure of different stress level of recommendations.

**Figure 10:** Accuracy measure of different positive emotion person of recommendations.

**Figure 11:** Precision measure of different positive emotion person of recommendations.

**Figure 12:** Recall measure of different positive emotion person of recommendations.

**Figure 13:** *F*1-measure of different positive emotion person of recommendations.

**Figure 14:** Precision measure of different negative emotion person of recommendations.

**Figure 15:** F1 measure of different negative emotion person of recommendations.

**Figure 16:** Accuracy measure of different positive thinking person of recommendations.

**Figure 17:** Precision measure of different positive thinking person of recommendations.

**Figure 18:** Recall measure of different positive thinking person of recommendations.

**Figure 19:** *F*1-measure of different positive thinking person of recommendations.

**Algorithm 1:** KNN Algorithm for grouping the similar set of users.

**Table 1:** Parameters of the recommender system.

User Id	Movie Id	Tag	Timestamp
2	60756	Funny	1.45*E* + 09
2	60756	Highly quotable	1.45*E* + 09
2	60756	Will Ferrell	1.45*E* + 09
2	89774	Boxing story	1.45*E* + 09
2	89774	MMA	1.45*E* + 09
2	89774	Tom Hardy	1.45*E* + 09
2	106782	Drugs	1.45*E* + 09
2	106782	Leonardo DiCaprio	1.45*E* + 09
2	106782	Martin Scorsese	1.45*E* + 09
7	48516	Way too long	1.17*E* + 09
18	431	Al Pacino	1.46*E* + 09
18	431	Gangster	1.46*E* + 09
18	431	Mafia	1.46*E* + 09
18	1221	Al Pacino	1.46*E* + 09

**Table 2:** Different types of participants and the Videos used by them.

S.No.	Type of participants	Type of contents	Number of users		
			Male	Female	Total
1	Sport videos watchers	Swimming, badminton, wrestling, Olympic shooting, cricket, football, tennis, hockey, ice hockey, kabaddi, gymnasium, weight lifting, volleyball, table tennis, baseball, Formula, MotoGP, chess, boxing, fencing, and basketball	5	2	7
2	Movie videos watchers	Action, comedy, drama, fantasy, horror, mystery, romance, thriller, and western	2	2	4
3	Social video watchers	Facebook, Instagram, Twitter, tutorials and how-to videos, product demo videos, user-generated videos, announcements/reveals, interview, and Q&A videos, event videos, behind-the-scenes, videos that promote exciting offers and deals, tell relatable stories, and final thoughts	2	4	6
4	Student/Learner videos watchers	Teaser videos and course videos	4	1	5
5	Medical/Professional/Business man content watchers	Surgery videos, Gynaecology and STDs, health and fitness, orthopaedics, cardiology, plastic surgery, medical examination, clinical skills, product videos, explainer videos, onboarding videos, internal training videos, testimonial videos, promotional videos, company culture videos. video voicemails, aerospace engineering videos, chemical engineering videos, electrical and electronics engineering videos, petroleum engineering videos, telecommunication engineering videos, machine learning and artificial intelligence videos, robotics engineering videos, and biochemical engineering videos.	6	2	8

The article "Sentiment Analysis of Statements on Social Media and Electronic Media Using Machine and Deep Learning Classifiers" was retracted in 2023. Reasons: signs of a paper mill; suspected computer-generated content; unreliable results or conclusions; concerns about the data.

**Table 3:** Average mobile interaction score.

S. No.	Type of watchers	Type of contents watched	Interaction score									
1	Sport videos watchers	Volleyball, cricket, football, tennis	45	50	55	60	65	70	75	80	85	90
			1	2	3	4	5	6	7	8	9	10
2	Movie videos watchers	Action, comedy, drama, fantasy, romance	10	20	30	40	50	60	70	80	90	100
			1	2	3	4	5	6	7	8	9	10
3	Social video watchers	Facebook, tutorials videos, Product demo videos, interview, and Q&A videos, event videos	6	8	10	12	14	16	18	20	22	24
			1	2	3	4	5	6	7	8	9	10
4	Student/Learner videos watchers	Teaser video, course videos	1–3				4–7			8–12		
			4				8			10		
5	Medical/Professional/Business man content watchers	Surgery videos, health and fitness, medical examination, clinical skills	1				2			3		
			4				8			10		

**Table 4:** Correlation between accuracy and other attributes.

Attribute 1	Attribute 2	Partial correlation
Accuracy (AC)	Hardness (HD)	0.882156
Accuracy (AC)	Stress (ST)	−0.51087
Accuracy (AC)	Positive emotion (PE)	0.42498
Accuracy (AC)	Negative emotion (NE)	−0.377452
Accuracy (AC)	Positive thinking (PT)	0.462025

## Data Availability

The data that support the findings of this study are available on request from the corresponding author.

## References

[1] Peter C., Beale R. (2008). Affect and emotion in human-computer interaction. *LNCS*.

[2] Jeon M. (2017). Emotions and affect in human factors and human-computer interaction: Taxonomy, Theories, approaches, and methods. *Emotions and Affect in Human Factors and Human-Computer Interaction*.

[3] Aday J., Rizer W., Carlson J. M. (2017). Neural mechanisms of emotions and affect. *Emotions and Affect in Human Factors and Human-Computer Interaction*.

[4] Elfenbein H. A., Sigal B., Noah E. C. (2015). Supplemental material for the social perception of emotional abilities: expanding what we know about observer ratings of emotional intelligence. *Emotion*.

[5] Kövecses Z. (2015). Happiness in context. *Where Metaphors Come From*.

[6] Ellis D., Tucker I. (2020). Artificial intelligence and emotion. *Emotion in the Digital Age*.

[7] Vallverdú J. (2016). Why robots must have synthetic emotions? The role of emotions in the artificial cognitive systems. *Proceedings*.

The article "Sentiment Analysis of Statements on Social Media and Electronic Media Using Machine and Deep Learning Classifiers" was retracted in 2023. Reasons: signs of a paper mill; suspected computer-generated content; unreliable results or conclusions; concerns about the data.

[8] Shen J., Rudovic O., Cheng S., Pantic M. Sentiment apprehension in human-robot interaction with NAO.

[9] Freed S. (2019). Prevailing Prejudices pertaining to artificial intelligence. *AI and Human Thought and Emotion*.

[10] Angeli A., Johnson G. (2003). Emotional intelligence in interactive systems. *Design and Emotion*.

[11] De Freitas J. S., Gudwin R., Queiroz J. Emotion in artificial intelligence and artificial life research: facing problems.

[12] Mahlke S., Minge M., Thüring M. Measuring multiple components of emotions in interactive contexts.

[13] Desmet P. (2018). Measuring emotion: development and application of an instrument to measure emotional responses to products. *Human-Computer Interaction Series*.

[14] Gupta R., Shukla P. K., Shukla P. K. (2015). Performance analysis of anti-phishing tools and study of classification data mining algorithms for a novel anti-phishing system. *International Journal of Computer Network and Information Security*.

[15] Ran S., Hsu S., Jung T. Examining the relationship between EEG dynamics and emotion ratings during video watching using adaptive mixture independent component analysis.

[16] Hsu S., Zi Y., Wu Y. C., Jackson P. M., Jung T. Exploring mental state changes during hypnotherapy using adaptive mixture independent component analysis of EEG.

[17] Tiwari P., Shukla P., Tuba M., Akashe S., Joshi A. (2020). Artificial neural network-based crop yield prediction using NDVI, SPI, VCI feature vectors. *Information and Communication Technology for Sustainable Development. Advances in Intelligent Systems and Computing*.

[18] Roy V., Shukla S., Shukla P. K., Rawat P. (2017). Gaussian elimination-based novel canonical correlation analysis method for EEG motion artifact removal. *Journal of Healthcare Engineering*.

[19] Bänziger T., Grandjean D., Scherer K. R. (2009). Emotion recognition from expressions in face, voice, and body: the multimodal emotion recognition test (MERT). *Emotion*.

[20] Sloman A. (1981). WHY robots will have emotions. *Proceedings IJCAI*.

[21] Pantic M. (2008). Human-centred intelligent human–computer interaction (HCI^2^): how far are we from attaining it?. *International Journal of Autonomous and Adaptive Communications Systems*.

[22] Khambra G., Shukla P. (2021). Novel machine learning applications on fly ash based concrete: an overview. *Materials Today Proceedings*.

[23] Smyth J. M. (1998). Written emotional expression: effect sizes, outcome types, and moderating variables. *Journal of Consulting and Clinical Psychology*.

[24] Yacoub S., Burns J., Lin X., Stevern S. J. Recognition of emotions in interactive voice response systems.

[25] Pandit S., Shukla P. K., Tiwari A., Shukla P. K., Dubey R. (2020). Review of video compression techniques based on fractal transform function and swarm intelligence. *International Journal of Modern Physics B*.

The article "Sentiment Analysis of Statements on Social Media and Electronic Media Using Machine and Deep Learning Classifiers" was retracted in 2023. Reasons: signs of a paper mill; suspected computer-generated content; unreliable results or conclusions; concerns about the data.

[26] Schröder M., Cowie R. (2006). Developing a consistent view on emotion-oriented computing. *Machine Learning for Multimodal Interaction*.

[27] Ashby F. G., Isen A. M., Turken A. U. (1999). A neuropsychological theory of positive affect and its influence on cognition. *Psychological Review*.

[28] Fredrickson B. L. (1998). what good are positive emotions?. *Review of General Psychology*.

[29] Nurkka P. User experience evaluation based on values and emotions.

[30] Shukla P. K., Kaur Sandhu J., Ahirwar A., Ghai D., Maheshwary P., Shukla P. K. (2021). Multiobjective genetic algorithm and convolutional neural network based COVID-19 identification in chest X-ray images. *Mathematical Problems in Engineering*.

[31] Kobasa S. C., Maddi S. R., Kahn S. (1982). Hardiness and health: a prospective study. *Journal of Personality and Social Psychology*.

[32] Manning C. D., Raghavan P., Schütze H. (2017). *Introduction to Information Retrieval*.

[33] Roy V., Shukla P. K., Gupta A. K., Goel V., Shukla P. K., Shukla S. (2021). Taxonomy on EEG artifacts removal methods, issues, and healthcare applications. *Journal of Organizational and End User Computing*.

[34] Fredrickson B. L. (2018). Biological underpinnings of positive emotions and purpose. *The Social Psychology of Living Well*.

